# Influence of Dexmedetomidine on Myocardial Injury in Patients with Simultaneous Pancreas-Kidney Transplantation

**DOI:** 10.1155/2022/7196449

**Published:** 2022-11-17

**Authors:** Aili Dong, Yajing Zhang, Shujun Lu, Wenli Yu

**Affiliations:** ^1^Tianjin First Center Hospital, Tianjin 300192, China; ^2^First Teaching Hospital of Tianjin University of Traditional Chinese Medicine, National Clinical Research Center for Chinese Medicine Acupuncture and Moxibustion, Tianjin 300193, China

## Abstract

**Background:**

Diabetes is one of the most common chronic diseases in the world. End-stage renal disease (ESRD) caused by diabetes is the most serious long-term complication. The main cause of death in patients with simultaneous pancreas-kidney transplantation (SPKT) is cardiovascular disease. Although dexmedetomidine (Dex) has unique advantages in heart protection against ischaemic/reperfusion injury, few clinical studies have been conducted on its cardioprotective effect in SPKT. This study aimed to explore the influence of Dex on myocardial injury in patients undergoing SPKT and to analyze its possible mechanism.

**Methods:**

A randomized controlled trial (RCT) was performed from July 1, 2018 to December 1, 2020. Eighty patients, regardless of gender, scheduled for SPKT were randomly allocated into a Dex group (D group) receiving Dex at a rate of 1 *µ*g/kg for 10 minutes before anaesthesia induction and then continuous infusion at 0.5 *µ*g/kg/hour until the end of surgery and control group (C group) receiving equivalent capacity of saline. Serum cardiac troponin I (cTnI), creatine kinase isoenzyme (CK-MB), tumour necrosis factor-*α* (TNF-*α*), and interleukin-6 (IL-6) were recorded at 5 minutes after anaesthesia induction (baseline,T0), 5 minutes before renal arteriovenous opening (T1), 30 minutes after renal arteriovenous opening (T2), 30 minutes after pancreatic related arteriovenous opening (T3), immediately after surgery (T4), 4 hours after surgery (T5), and 24 hours after surgery (T6). Adverse cardiovascular events were recorded during the perioperative period. Changes in ECG S-T segments and *T* waves were monitored at T0–T6. Myocardial infarction and percutaneous coronary intervention were recorded with an average follow-up of one year.

**Results:**

Compared with T0, TNF-*α* and IL-6 concentrations significantly increased at T1–T6 in the C and D groups (*P* < 0.05). IL-6 concentration increased significantly after renal artery opening and reached the peak after the opening of pancreatic blood vessels. Compared with the C group, TNF-*α*, and IL-6 concentrations were significantly reduced in group D at T2–T6 (*P* < 0.05). Compared with T0, cTnI and CK-MB concentrations were significantly increased at T3–T6 in the C and D groups (*P* < 0.05). cTnI and CK-MB concentrations increased significantly after the opening of renal artery, and reached the peak after the opening of pancreatic blood vessels. Compared with the C group, cTnI and CK-MB concentrations were significantly reduced in the D group at T3–T6 (*P* < 0.05). There was no significant difference in patient characteristics amongst groups, including the proportion of intraoperative vasoactive drug use and adverse cardiovascular events during the follow-up period. Heart rate, mean blood pressure, central venous pressure, and cardiac output were not remarkably different between the two groups at any time point.

**Conclusions:**

Perioperative reperfusion could aggravate myocardial injury in SPKT. Dex may be considered a way to reduce myocardial injury caused by inflammatory action by decreasing the release of inflammatory factors. Trial Registration Number: Chinese Clinical Trial Registry ID: ChiCTR2200060084.

## 1. Introduction

Diabetes is one of the most common chronic diseases in the world. End-stage renal disease (ESRD) caused by diabetes is the most serious long-term complication. About 30% of patients die from renal failure [1]. The incidence rate of diabetic nephropathy is 50%–60%, and the probability of diabetic nephropathy is increasing with age and duration. Pancreas transplantation is one of the most important way to cure diabetes. It can provide insulin replacement therapy for diabetic patients [2]. Simultaneous pancreas transplantation is an effective method for the treatment of type 1 diabetes mellitus (T1DM) with ESRD and type 2 diabetes mellitus (T2DM) with renal failure [3–5]. The survival time of patients undergoing simultaneous pancreas-kidney transplantation (SPKT) is longer than those of patients who have kidney transplantation alone [6].

The main cause of death in patients with SPKT is cardiovascular disease(CV) [7]. As diabetes accelerates atherosclerosis, it can have a serious impact on the cardiovascular system. If ESRD is complicated at the same time, the cardiovascular risk will be greatly increased [8]. Therefore, reducing the incidence of perioperative adverse cardiovascular events and enhancing cardiac protection are of great importance for the success of surgery and the prognosis of patients.

As a highly selective *α*2-adrenergic receptor (*α*2-AR) agonist, dexmedetomidine (Dex) has sedative and analgesic effects, and inhibits sympathetic excitation and is widely used in cardiac anaesthesia. Dex is characterized by quick distribution into the tissues together with a short half-life and adverse effects are few in number, mild in severity [9]. It can effectively inhibit abnormally increased blood pressure and heart rate under stress, stabilise haemodynamics, reduce myocardial ischaemia, improve the prognosis of patients, and have myocardial protection by reducing the sympathetic nerve activity [10].

Although Dex is effective in protecting human cardiocytes from ischaemia-reperfusion (I/R) injury in vivo and hypoxia-reoxgenation (H/R) injury in vitro [11–13], few clinical studies have been conducted on its cardioprotective effect in SPKT and its mechanism. In the preliminary research, we observed changes in inflammatory indexes, such as pro-inflammatory cytokines Interleukin 6 (IL-6)and TNF-*α* in SPKT, which began to rise after the opening of the pancreatic artery, suggesting the presence of an organ injury in patients with SPKT. Therefore, this study aimed to explore the cardioprotective effect of Dex in SPKT and the possible mechanism through changes in haemodynamic parameters and the correlation between the balance of pro-inflammatory and anti-inflammatory factors. This can provide relevant reference to fill the clinical gap in the influence of Dex on myocardial injury in patients with SPKT.

## 2. Methods

### 2.1. Participants

This research was approved by Institutional Ethics Committee of Tianjin First Center Hospital (approval no.2018N110KY). The patients were recruited between July 1, 2018 and December 1, 2020. Eighty patients with DM and ESRD were scheduled for renal and pancreatic allograft from deceased donors. The patients enrolled in this trial were American Society of Anaesthesiologists (ASA) II–IV aged 18–60 years with no severe heart failure and serious liver and pulmonary dysfunction. All transplants were performed by homolateral simultaneous pancreas–kidney transplantation with systemic venous drainage and enteric drainage of exocrine secretions. The exclusion criteria were: (I) patients with known or suspected allergy to Dex; (II) patients who needed renal and/or pancreatic transplantation after operation; (III) patients with a history of cognitive disorder or on any psychotropic medication at the time of the study; (IV) patients with a history of serious arrhythmia, such as remarkable bradycardia and 3rd degree atrioventricular block or (V) impairment of liver and/or pulmonary function before SPKT. The study was approved by the institutional ethics committee, and all patients or authorised family members gave written informed consent.

### 2.2. Anaesthesia and Design

The patients enrolled in this study were randomly and equally divided into the Dex group (D group) and control group (C group) using a random number table. All patients were randomly assigned to the groups by a computer-generated random number system individually sealed in envelopes. Patients were blinded to the group assignment. Another anaesthesiologist was responsible for data collection but not directly involved in the treatment of patients and blinded to randomisation. In the D group, patients received a loading dose of Dex (Batch number: 22012131, Jiangsu Nhwa Pharmaceutical Co., Ltd. China) at a rate of 1 *µ*g/kg for 10 minutes before anaesthesia induction and then received a continuous infusion at 0.5 *µ*g/kg/hour until the end of surgery. The control group received an equivalent capacity of saline at the same time point.

The patients were instructed to fast and abstain from beverages before surgery. After entry into the operating room, a peripheral venous passage was established and electrocardiogram (ECG), blood pressure, blood oxygen saturation, bispectral index, and heart rate (HR) were monitored continuously throughout the surgery. All patients received general anaesthesia with tracheal intubation. Midazolam (0.05 mg/kg) and atropine (0.3 mg) were injected. An arterial pressure monitoring catheter was implanted after radial artery puncture. Right internal jugular vein cannulation was accomplished using a Doppler ultrasound instrument. Cardiac output (CO) was monitored by FloTrac/Vigileo throughout the operation, as well as invasive radial arterial pressure and central venous pressure (CVP). Anaesthesia induction was performed with 1-2 mg/kg propofol, 1 *μ*g/kg sufentanil, and 0.15 mg/kg cisatracurium besylate. For anaesthesia maintenance, 6–10 mg/kg/hour propofol and 0.02–0.2 mg/kg/hour remifentanil were used during surgery. Sevoflurane (1%–2%) was also used with the minimal effective concentration for anaesthesia.

Maintaining circulatory stability and achieving mean arterial pressure (MAP) ≥ 90 mmHg are necessary to sustain organ perfusion before the opening of the renal artery and pancreatic artery by infusing dopamine. Patients receiving prudent strategies for fresh refrigerated plasma and clotting factor transfusion should be monitored closely for coagulation function. Basiliximab (10 mg) combined with methylprednisolone (500 mg/day) were routinely administered for immune induction after the opening of the renal artery. Aprotinin (0.1 mg) was injected subcutaneously to inhibit trypsin and chymotrypsin and prevent intestinal mucosal injury before the opening of the pancreatic artery. Metronidazole (50 mg) was injected intravenously to prevent the disturbance of intestinal microbiota. If bradycardia occurred, application of atropine could be effectively alleviated in general.

### 2.3. Blood Assays

Central venous blood (6 mL) samples were collected, and the concentrations of serum cardiac troponin I (cTnI), creatine kinase isoenzyme (CK-MB), tumour necrosis factor-*α* (TNF-*α*), interleukin-6 (IL-6), and interleukin-18 (IL-18) were recorded at the following times: 5 minutes after anaesthesia induction (baseline,T0), 5 minutes before renal arteriovenous opening (T1), 30 minutes after renal arteriovenous opening (T2), 30 minutes after pancreatic related arteriovenous opening (T3), immediately after surgery (T4), 4 hours after surgery (T5), and 24 hours after surgery (T6).

### 2.4. Data Collection

The following patients and preoperative variables were included: patient characteristics, such as age, gender, body mass index (BMI), type of diabetes, duration of diabetes, dialysis duration pretransplant, and graft cold ischaemia time. Intraoperative data, including the proportion of intraoperative vasoactive drug use, operation time, bleeding volume, blood transfusions, and urine volume were collected. Postoperative data, including extubation time, intensive care unit (ICU) stay time, and hospitalisation, were collected. Adverse cardiovascular events were recorded during the perioperative period. Changes in ECG S-T segments and *T* waves were monitored at T0–T6, and the number of intraoperative circulating perfusion, hypertension, or hypotension (blood pressure increased or decreased by 30% or more from the baseline value for more than 10 minutes), myocardial ischaemia (ST segment depression or elevation greater than 1 mm and lasting longer than 1 minute), and ventricular premature beats were recorded.

### 2.5. Statistical Analysis

Statistical analyses were performed by SPSS21.0 (SPSS Inc, Chicago, IL, USA). Kolmogorov–Smirnov was used to analyze the data distribution. Continuous and categorical variables were reported as mean (standard deviations), medians (interquartile ranges), or percentages. Patient characteristics and perioperative clinical data in the two groups were compared by using independent *t*-test or Fisher's exact test, as appropriate. Group comparisons of haemodynamic variables and myocardial injury biomarkers at each time point were analyzed by using an independent *t*-test. Changes in group haemodynamic variables and myocardial injury biomarkers over time were analyzed by using ANOVA followed by appropriate post hoc test. Comparison of count data was used with *χ*^2^ test or Fisher's exact test. *P* < 0.05 was considered statistically significant.

## 3. Results

### 3.1. Patient Characteristics and Intraoperative Data

The study flow is depicted in Figure 1.  Table 1 lists the patient characteristics. Total operative times, bleeding volume, and urine volume, as well as blood transfusions, extubation time, ICU time, and hospitalisation time, were similar in both groups. Similarly, no remarkable differences in adverse cardiovascular events and the proportion of intraoperative vasoactive drug use were observed between the two groups.

### 3.2. Perioperative Haemodynamic Changes

The haemodynamic variables are presented in Table 2. HR, MAP, CVP, and CO were not remarkably different between the two groups at any time point.

### 3.3. Differences of Inflammatory Factors and Myocardial Injury Biomarkers

TNF-*α* and IL-6 concetrations are shown in Figures 2 and 3. Compared with T0, TNF-*α* and IL-6 concentrations significantly increased at T1–T6 in the C and D groups (*P* < 0.05). IL-6 concentration increased remarkably after the opening of the renal artery and reached the peak after the opening of pancreatic blood vessels. Compared with the C group, TNF-*α* and IL-6 concentrations were significantly reduced in the D group at T2–T6 (*P* < 0.05).

Changes in cTnI and CK-MB are shown in Table 3 and4. Compared with T0, cTnI and CK-MB concentrations were significantly increased at T3–T6 in the C and D groups (*P* < 0.05). cTnI and CK-MB concentrations increased remarkably after the opening of the renal artery and reached the peak after the opening of pancreatic blood vessels. Compared with the C group, cTnI and CK-MB concentrations were markedly reduced in the D group at T3–T6 (*P* < 0.05).

### 3.4. Intraoperative Adverse Cardiovascular Events

Twenty-one patients (52%) in the C group and 16 patients (40%) in the D group showed S-T segment depression or T wave apex at T2, and 23 patients (58%) in the C group and 17 patients (43%) in the D group showed S-T segment depression or T wave apex at T3. Fourteen patients (35%) in the C group and ten patients (25%) in the D group needed intravenous dopamine infusion to maintain circulatory perfusion. The incidence rates of hypertension or hypotension, myocardial ischaemia, and premature ventricular beats showed no statistical differences between the two groups.

## 4. Discussion

The cardiovascular system of patients with end-stage diabetes nephropathy is damaged in varying degrees, in which the main clinical manifestations are myocardial injury caused by the metabolic and haemodynamic changes resulting in cardiac systolic or diastolic dysfunction and coronary artery disease. Additionally, patients with varying degrees of hypertension and autonomic nerve fibre disease have an increased risk of asymptomatic myocardial ischaemia or even myocardial infarction during the perioperative period, as well as other adverse cardiovascular complications [14]. Cardiovascular system impairment threatens patient survival and increases the risk of the perioperative period.

Amongst patients with ESRD and T1DM, SPKT is the preferred method for kidney and pancreatic replacement therapy. The successful implementation of SPKT tends to restore optimal glycaemic control and therefore stabilises the secondary complications associated with T1DM [15]. As a result, it increases the life expectancy of patients and their quality of life by slowing the progression of CV [16, 17]. However, SPKT is a complex procedure that triggers an inflammatory response and activates the sympathetic nervous system, which may potentially cause cardiac injuries. Additionally, plenty of free radicals activate inflammatory cells following reperfusion, which give rise to cell membrane damage and increased permeability. This process causes myocardial metabolic disturbance, structural damage, and functional disorder [18]. Our study found that cTnI and CK-MB concentrations began to increase substantially after renal I/R in the two groups and peaked after pancreatic I/R. cTnI and CK-MB concentrations were still high 24 hours postoperatively and were remarkably higher than those in the preoperative stage, suggesting that various degrees of myocardial injury are present from the intraoperative period to the postoperative period.

Cardiocytes are nucleated cells in the myocardium that can secrete pro-inflammatory cytokines in response to myocardial stress or injury [19]. IL-6 and TNF-*α* have relevance to functional New York Heart Association (NYHA) class in systolic heart failure [20]. In addition, IL-6 and TNF-*α* serve as independent predictors of mortality in patients with heart failure [21]. Lianza et al. [22] found that left ventricular structure and function improved remarkably by repressing serum IL-6 and TNF-*α* levels. Plenz et al. [23] showed that IL-6 level considerably affected ventricular function in different cardiac functional states for living donors with heart transplantation. Increased IL-6 levels in the myocardium could lead to cardiac dysfunction. Therefore, Dex can improve cardiac function, reduce postoperative cardiac complications, and promote the success rate of surgery by reducing the level of IL-6 in heart transplantation. TNF-*α* can cause cardiomyocyte injury by inducing the overexpression of nitric oxide synthase in cardiomyocytes [24]. The results of our study showed that the rising time points of serum TNF-*α* and IL-6 at the intraoperative and postoperative periods were slightly earlier than those of myocardial injury markers. The peak time point appeared at the same time, suggesting that the excessive release of a large number of inflammatory cytokines may be an important factor causing myocardial injury.

In recent years, more basic and clinical studies have found that Dex has unique advantages in the protection of multiple organs, such as the brain, heart, liver, kidney, and lung [13, 25, 26]. Dex is an alpha2 adrenoceptor agonist that inhibits inflammatory mediator production and decreases cell death, apoptosis, and necroptosis [27]. Considering the importance of inflammation and apoptosis, as well as potential anti-inflammation and apoptosis effects [28], Dex has been widely used in perioperative anaesthesia maintenance as an effective organ protective agent. Dex remarkably reduces the incidence of perioperative cardiovascular complications, such as myocardial infarction, in patients undergoing coronary artery bypass grafting [29]. Dex also exerts a cardioprotective effect against heart ischaemia in vitro, which is mediated by *α*2-adrenergic stimulation [30]. Huang et al. [31] found that the hepaprotective effect of Dex appears to involve the attenuation of oxidative stress and the inhibition of inflammatory response, which play crucial roles in hepatic IR injury. Dex can attenuate inflammatory cytokines, such as TNF and IL-6, by inhibiting the activation of extracellular regulated protein kinases1/2(ERK1/2) and NF-*κ*B, modulating inflammatory mediators, reducing the systemic inflammatory response, and improving the outcomes in kidney transplantation [32]. Xiao [12] et al. demonstrated that Dex is effective in human heart I/R injury protection, and *α*2-adrenergic receptor/AMP-activated protein kinase (AMPK)-dependent autophagy may be one of the mechanisms by which Dex protects human heart tissues from I/R injury. This result was consistent with our findings that the levels of serum IL-6 and TNF-*α* were notably increased after the opening of the renal artery and peaked after the opening of the pancreatic artery. Compared with the C group, the concentrations of IL-6 and TNF-*α* were remarkably reduced in the D group after the opening of the renal artery until post-operation, suggesting Dex may attenuate systemic inflammatory response by inhibiting the release of inflammatory factors in SKPT.

Additionally, Dex blunts haemodynamic responses to perioperative stress, properly controls the heart rate, and optimises the blood flow in coronary arteries by blocking the sympathetic nervous system [30]. Despite the lack of statistical significance, the haemodynamics in the Dex group tend to be more stable than that in control group at the time of reperfusion. Most of the time, transient blood pressure reduced at the time of reperfusion. Vasoactive drugs, such as dopamine and norepinephrine, were used to increase blood pressure so that the blood pressure was reduced by no longer than 2 minutes. No differences in the proportions of intraoperative vasoactive drug use were found between the two groups.

cTnI and CK-MB are the markers used for the early diagnosis of myocardial injury in clinics. Serum cTnI and CK-MB concentrations increased at 4–6 hours after myocardial injury and reached the peak at 12–24 hours [33]. cTnI exists only in cardiomyocytes and is the most sensitive index for predicting and diagnosing myocardial injury [34]. The ECG manifestations of myocardial injury include *T* wave high peak, S-T segment elevation or reduction, acute traumatic conduction block, and ischaemic *g* wave. Many factors influence ECG performance and the lack of specificity [35]. This study can help evaluate the degree of cardiomyocyte injury by analysing the indexes above. Deng et al. found that Dex preconditioning exerted a cardioprotective effect against regional I/R injury in diabetic rats [36], Ammar et al. revealed that Dex provides some degree of heart protection during cardiac surgery as evidenced by the lower levels of myocardial-specific proteins (cTnI and CK-MB) and combined with lower levels of serum pro-inflammatory cytokines (TNF-*α* and IL-1*β*) [37]. Similar to our results, the concentrations of serum cTnI and CK-MB increased gradually after renal vascular opening in the two groups. The application of Dex considerably decreased cTnI and CK-MB concentrations. Moreover, ECG monitoring showed that the incidence of myocardial injury was also reduced, suggesting that Dex has a certain protective effect on myocardial injury.

In this study, ECG monitoring showed that myocardial injury occurred after the opening of renal and pancreatic vessels with incidence rates of 48% and 56%, respectively. The incidence of intraoperative adverse cardiovascular events was 24%, which were manifested by hypotension and myocardial ischaemia. The compensatory ability of the heart to the change in intravascular volume decreased, which easily caused the instability of perioperative circulatory function. Many of the patients with ischaemic heart disease had no conscious symptoms. Therefore, cardiovascular function should be strictly evaluated before operation, and the monitoring and management during operation should be strengthened to improve the perioperative safety. The use of Dex in this study did not reduce the incidence of adverse cardiovascular events, which may be related to the long-term damage of the cardiovascular system in patients with end-stage diabetes nephropathy and the small sample size of the study.

The primary limitations of this study are as follows: (1) This single-centre trial has a small sample size. A multicentre clinical research with a large sample is needed in the later stage; (2) The research mechanism and other influencing factors of Dex on myocardial protection in these patients need to be further studied and discussed; (3) Dex is dose dependent in the scope of routine use and time dependent in the maximum anti-inflammatory response. The optimal dose, action time, and treatment scheme in myocardial protection need to be further studied; (4) The long-term survival rate of patients after operation needs to be studied, and whether the application of Dex can affect the survival rate of grafts and patients should be explored.

In conclusion, as far as we know, the current study firstly demonstrated the influence of Dex on myocardial injury in patients with SPKT. Perioperative reperfusion can aggravate the myocardial injury, and Dex may be considered a way to reduce the myocardial injury of inflammatory action by decreasing the release of inflammatory factors.

## Figures and Tables

**Figure 1:** Patient population. Five of the 99 patients who underwent SPKT were excluded because of age limitation. The remaining 94 patients were randomly divided into the Dex and control groups. Amongst these patients, 14 patients were excluded for repeated operations and lost to follow-up. Thus, 80 patients were included in the final analysis (*n* = 40, each).

**Figure 2:** TNF-*α* trends at every time point. Values are presented as mean ± SD. T0: 5 minutes after anaesthesia induction; T1: 5 minutes before renal arteriovenous opening; T2: 30 minutes after renal arteriovenous opening; T3: 30 minutes after pancreatic related arteriovenous opening; T4: immediately after surgery; T5: 4 hours after surgery; T6: 24 hours after surgery.  ^*∗*^*P* < 0.05 compared with C group, ^#^*P* < 0.05 compared with T0. TNF-*α*, tumour necrosis factor-*α*.

**Figure 3:** IL-6 trends at every time point. Values are presented as mean ± SD. T0: 5 minutes after anaesthesia induction; T1: 5 minutes before renal arteriovenous opening; T2: 30 minutes after renal arteriovenous opening; T3: 30 minutes after pancreatic related arteriovenous opening; T4: immediately after surgery; T5: 4 hours after surgery; T6: 24 hours after surgery.  ^*∗*^*P* < 0.05 compared with C group, ^#^*P* < 0.05 compared with T0. IL-6, interleukin-6.

**Table 1:** Patient demographic and perioperative data.

Variables	C Group	D group	t/*χ*^2^	*P*
Age at transplantation (years)	45.6 ± 8.5	46.4 ± 9.7	0.367	0.714
Gender (boy/girl, (*n*))	29/11	26/14	0.524	0.469
BMI (kg/m^2^)	24.3 ± 3.5	23.8 ± 3.7	0.616	0.540
Duration of diabetes (years)	13.8 ± 5.1	14.1 ± 6.0	0.222	0.825
Type of diabetes (type1/type2, (*n*))	9/31	7/33	0.313	0.576
Dialysis duration pretransplant (months)	27.0 (23–38)	25.5 (21–30)	1.151	0.250
Operation time (min)	461.3 ± 65.2	451.8 ± 51.1	0.725	0.470
Bleeding volume (mL)	300 (250–387)	325 (250–400)	1.210	0.226
Intraoperative blood transfusions (U)	4.0 (2.0–5.0)	4.0 (2.0–4.5)	0.074	0.941
Urine volume (mL)	657.3 ± 223.6	665.9 ± 251.5	0.164	0.870
Graft cold ischaemia time (h)	4.9 ± 1.1	4.8 ± 1.0	0.221	0.825
Proportion of intraoperative vasoactive drug use (%)	8 (20)	11 (28)	0.621	0.431
Extubation time (min)	217.5 ± 76.4	230.6 ± 65.0	0.828	0.410
ICU time (d)	6.0 ± 2.1	5.6 ± 3.4	0.852	0.397
Hospitalisation time (d)	25.1 ± 5.9	27.6 ± 8.2	1.522	0.133

Values are presented as mean ± SD, medians (interquartile ranges), or number of patients (%). ASA, American Society of Anesthesiologist; BMI, body mass index; ICU, intensive care unit.

**Table 2:** Changes in haemodynamic variables at every time point.

Variables	Group	*T*_0_	*T*_1_	*T*_2_	*T*_3_	*T*_4_	*T*_5_	*T*_6_
HR (bpm)	C group	79.5 ± 14.0	83.5 ± 9.2	82.0 ± 12.3	82.3 ± 10.2	80.2 ± 11.9	80.4 ± 12.9	84.4 ± 9.3
	D group	81.5 ± 12.7	86.5 ± 9.9	83.6 ± 13.0	78.6 ± 10.7	82.1 ± 11.2	81.0 ± 9.1	80.7 ± 12.0

MAP (mmHg)	C group	101.8 ± 13.1	103.0 ± 9.2	99.1 ± 5.8	104.4 ± 10.6	101.9 ± 10.7	92.4 ± 6.8	95.7 ± 7.0
	D group	104.0 ± 13.2	107.4 ± 11.8	97.8 ± 6.7	102.0 ± 9.9	99.7 ± 10.7	95.3 ± 8.2	98.2 ± 4.9

CVP (mmHg)	C group	6.1 ± 2.5	9.0 ± 2.1	8.0 ± 1.6	8.4 ± 1.3	8.1 ± 1.8	7.6 ± 1.3	5.7 ± 2.0
	D group	5.8 ± 1.7	8.8 ± 1.5	7.9 ± 1.5	8.2 ± 1.5	7.9 ± 1.6	7.5 ± 1.9	6.2 ± 1.8

CO (L/min)	C group	4.8 ± 0.7.	6.0 ± 0.8	6.9 ± 0.8	5.9 ± 0.8	4.9 ± 0.6	4.8 ± 0.7	4.6 ± 0.6
	D group	4.6 ± 0.8	5.9 ± 0.9	6.8 ± 0.9	6.1 ± 0.7	4.9 ± 0.7	4.9 ± 0.6	4.8 ± 0.6

Values are presented as mean ± SD. T0: 5 minutes after anaesthesia induction; T1: 5 minutes before renal arteriovenous opening; T2: 30 minutes after renal arteriovenous opening; T3: 30 minutes after pancreatic related arteriovenous opening; T4: immediately after surgery; T5: 4 hours after surgery; T6: 24 hours after surgery.  ^*∗*^*P* < 0.05 compared with control, ^#^*P* < 0.05 compared with T0. MAP, mean arterial blood pressure; HR, heart rate; CVP, central venous pressure; CO, cardiac output.

**Table 3:** Changes in myocardial injury biomarkers at every time point.

Variables	Control group		Dex group	
	cTnI (*μ*g/L)	CK-MB (*μ*g/L)	cTnI (*μ*g/L)	CK-MB (*μ*g/L)
T0	0.05 ± 0.01	1.64 ± 0.30	0.05 ± 0.01	1.65 ± 0.32
T1	0.06 ± 0.00^#^	1.99 ± 0.37^#^	0.05 ± 0.01^#^	2.04 ± 0.37^#^
T2	0.20 ± 0.03^#^	5.74 ± 0.39^#^	0.09 ± 0.01^#^ ^*∗*^	3.25 ± 0.49^#^ ^*∗*^
T3	0.32 ± 0.02^#^	7.76 ± 0.35^#^	0.17 ± 0.01^#^ ^*∗*^	4.84 ± 0.29^#^ ^*∗*^
T4	4.84 ± 0.29^#^ ^*∗*^	10.88 ± 0.49^#^	0.32 ± 0.04^#^ ^*∗*^	7.35 ± 0.32^#^ ^*∗*^
T5	0.50 ± 0.01^#^	9.50 ± 0.55^#^	0.17 ± 0.01^#^ ^*∗*^	5.88 ± 0.30^#^ ^*∗*^
T6	0.43 ± 0.01^#^	7.46 ± 0.33^#^	0.17 ± 0.01^#^ ^*∗*^	4.61 ± 0.18^#^ ^*∗*^

Values are presented as mean ± SD. T0: 5 minutes after anaesthesia induction; T1: 5 minutes before renal arteriovenous opening; T2: 30 minutes after renal arteriovenous opening; T3: 30 minutes after pancreatic related arteriovenous opening; T4: immediately after surgery; T5: 4 hours after surgery; T6: 24 hours after surgery.  ^*∗*^*P* < 0.05 compared with C group, ^#^*P* < 0.05 compared with T0. cTnI, cardiac troponin I; CK-MB, creatine kinase isoenzyme.

**Table 4:** Incidence rates of adverse cardiovascular events at different time points.

Variables	C Group	D group	*P*
Cardiovascular events pretransplant			
Myocardial infarction	3 (7.5)	4 (10)	0.231
Percutaneous coronary intervention	7 (17.5)	9 (22.5)	0.064
Coronary artery bypass graft	2 (5)	1 (2)	0.938

Adverse intraoperative cardiovascular events			
Hypertension	5 (12)	3 (8)	0.456
Hypopiesia	3 (8)	4 (10)	0.694
Ischaemia myocardial	1 (2)	0 (0)	0.314
Premature ventricualr contraction;	2 (5)	1 (2)	0.556

Cardiovascular events occurring one year after SPKT			
Myocardial infarction	2 (5)	0 (0)	0.152
Percutaneous coronary intervention	0 (0)	1 (2)	0.311

## Data Availability

Raw data associated with this article are provided in the supplementary material including patient data, haemodynamic parameters, and serum indexes.

## Supplementary Materials

Supplementary Materials The patient data, haemodynamic parameters, and serum indexes.
